This article has been retracted.

# Comparative Analysis of Antioxidants Activity of Indigenously Produced *Moringa Oleifera* Seeds Extracts

**DOI:** 10.1155/2022/4987929

**Published:** 2022-10-15

**Authors:** Sadaf Tariq, Huma Umbreen, Razia Noreen, Cyril Petitbois, Kiran Aftab, Fatmah Ali Alasmary, Amani Salem Almalki, Mohammad Abdul Mazid

**Affiliations:** ^1^Department of Biochemistry, Government College University Faisalabad, Pakistan; ^2^Department of Nutritional Sciences, Biochemistry, Government College University, Faisalabad, Pakistan; ^3^Inserm U1029 LAMC Group « 3D' Spectro-Imaging », University of Bordeaux, 33600 Pessac, France; ^4^Department of Chemistry, Government College University Faisalabad, Pakistan; ^5^Chemistry Department, College of Science, King Saud University, Riyadh 11451, Saudi Arabia; ^6^Department of Pharmaceutical Chemistry, Faculty of Pharmacy, University of Dhaka, Dhaka 1000, Bangladesh

## Abstract

Medicinal plants are used to control and remediate oxidative stress related diseases caused by free radicals. Thus, these plants find their use as remedy. *Moringa oleifera* is an extremely valued plant for its medicinal properties. Herein, two indigenously produced accessions of *Moringa oleifera* seeds [originated from Multan (M-Mln) and India (PKM1)] were investigated for their antioxidant properties by 2.2-Diphenyl-1picrylhydrazyl (DPPH) assay, total phenolics content and total flavonoids content. The presence of various phenolics as well as flavonoids was further confirmed by high performance liquid chromatography. Moreover, fourier transform infrared spectroscopy detected the presence of various functional groups. In conclusion, these findings revealed that the methanol extract of M-Mln variety seeds showed high antioxidant potential, having IC50 value of 84 *μ*g/ml. While, hexane extract of PKM1 showed least activity. The methanol extract of M-Mln was found to show highest total phenolics content as 33.83 ± 1.19 mg GAE/g. The methanol extract of M-Mln was found to show highest total flavonoids content as 76.07 ± 1.10 mg CAE/g. The hexane extract of PKM1 was found to show least total flavonoids content as 22.47 ± 1.70 mg CAE/g. The detection of phenolics (ferulic acid, caffeic acid, chlorogenic acid, coumaric acid, and gallic acid) as well as flavonoids (catechin and quercetin) revealed the potential of methanol extracts of both varieties as a good source of antioxidants. The results indicated the importance of seed extracts in the treatment of oxidative stress related diseases. In future, the use of natural antioxidants will prevent the progression of diseases.

## 1. Introduction

In living systems, oxidation reactions occur commonly. The cellular metabolism and respiration are reactions which frequently occur in human body. These oxidation reactions produce free radicals, such as reactive oxygen species as well as reactive nitrogen species [1]. These free radicals not only initiate different chain reactions, often toxic to cells, but also cause several destructive effects such as lipid peroxidation, DNA damage, protein degradation, and tissue injury which contribute to different diseases such as arthritis, liver diseases, atherosclerosis, diabetes, cancer, neurodegenerative disorders, and ageing [2, 3]. The detrimental effects of free radicals cause potential biological damage in living cells, also known as oxidative stress, when production of free radicals is overwhelmed by the body's ability to defend against free radicals [4, 5].

The human body is naturally blessed with different antioxidants (i.e., enzymatic and nonenzymatic) as defensive mechanism like thioredoxin, superoxide dismutases, catalases, uric acid, glutathione, and ascorbic acid which help the body to terminate the chain reactions initiated by free radicals [6, 7]. Nowadays, there is an increased interest in natural antioxidants that may be used to oppose free radicals with a view to lower the risk of associated diseases. Such reservoirs of natural antioxidants are different products of plant origin [4, 8].

*Moringa oleifera* (*M. oleifera*) is a small sized shrub like deciduous tree with soft and fragile stem found in different regions of the world, which belongs to family Moringaceae, native to Pakistan, India, Pacific Island, South America, Africa, Arabian Peninsula, Southeast Asia, and Caribbean Islands [1, 2]. It is grown in tropics and subtropics regions of the world. Because it is being cultivated in different regions of the world, *M. oleifera* is also known by many other local names i.e., horseradish tree, miracle tree, drumstick tree, and ben oil tree [9]. Due to its excessive use at household, it is commonly called as “The Mother's Best Friend”. A number of therapeutics and various medicinal characteristics have been attributed to different parts of tree due to presence of minerals and vitamins. Moringa species contain numerous unique compounds and it contains compounds rich in rhamnose, a simple carbohydrate. Glucosinolates and isothiocyanates, a group of compound is characteristically found in moringa family.

Specific parts of Moringa are reported to have 4-(4′O acetyl rhamnopyranosyloxy) benzyl isothiocyanate, an effective antibacterial agent (Bhattacharya et al.), pterygospermin, benzyl isothiocyanate [10], 4 (L-rhamnopyranosyloxy) benzyl glucosinolate [11], 4 (L-rhamnopyranosyloxy) benzyl isothiocyanate [12], and niazimicin as effective hypotensive and anticancer agents [13]. *M. oleifera* plant have potent antimicrobial, aphrodisiac, antihyperglycemic, antiulcer, antioxidant, antiepileptic, anticancer, antihypertensive, and anti-inflammatory activities (Asmari et al.) as listed in Table 1. The hypotensive, antibacterial, and anticancer activity is reported in seeds extracts due to some specific components as 4-(4′-acetyl rhamnopyranosyloxy)benzyl isothiocyanate, benzyl isothiocyanate, niazimicin, and pterygospermin [14, 15]. It is a source of polyphenols which are reported for antioxidant, antimicrobial, anticancer, anti-inflammatory, antihypertensive, antitumor, and antifungal activity. Some of the most reported phytochemical compounds are flavonoids, luteolin, quercetin, tannins, triterpenes, and glycosides. The antioxidant activity varies with environmental conditions, plant tissues, and harvest season [16, 17].

The seeds of the plant exhibit various biological activities like, antidiabetic [31], anti-inflammatory [32], hepatoprotective [33], anticancer [34], cardiovascular, CNS, analgesic [35], wound healing [36], antiallergic, antifertility, antiasthmatic [37], antiulcer, and antipyretic activity [38]. Therefore, this study was designed to evaluate the antioxidant potential of *M. oleifera* seeds of two different accessions from different regions. This study quantified the polyphenolic contents (i.e., total phenolics and total flavonoids) and estimated phytochemicals to investigate free radical scavenging activity *viz a viz* the antioxidant activity of various extracts of *M. oleifera* Multan (M-Mln) and Indian (PKM1) variety seeds.

## 2. Materials and Methods

### 2.1. Plant Material and Extraction

The seeds of *M. oleifera* of two different accessions, originated from Multan (M-Mln) and India (PKM1) were collected from *M. oleifera* plants grown at Department of Crop Physiology, University of Agriculture, Faisalabad, Pakistan. The seeds were authenticated by the Faculty of Department of Botany, Government College University, Faisalabad, Pakistan. Prior to extraction, the seed wings and coats were removed manually and the obtained kernels were ground in blender to obtain fine powder. The powder of both varieties were extracted with 100% methanol and n-Hexane. It was filtered by Whatman No. 1 filter paper. The excess solvent was evaporated at 40°C in a rotary evaporator and it was concentrated to crude extract and it was kept at 4°C in air tight dark bottles. The sample and solvent mass ratio was kept at 1 : 10 during extraction.

### 2.2. Fourier Transform Infrared Spectroscopy

FTIR spectroscopy (Perkin Elmer, USA) was done to evaluate the presence of various compounds and functional groups through ATR sampling technique in % transmittance mode (in the range of 4000-500 cm^−1^) with 45 scan recorder [39]. Dry powder of *M. oleifera* seeds was used for FTIR analysis. 10 mg of dry powder was encapsulated in 100 mg of potassium bromide pellets. The samples were loaded in FTIR spectrophotometer, and recorded spectra was obtained.

### 2.3. High Performance Liquid Chromatography

HPLC was performed in accordance with chromera HPLC system (Perkin Elmer, USA). HPLC was done to estimate different phenolics and flavonoids in methanol seed extracts of both varieties [40]. The sample was prepared by dissolving 50 mg of extract in 40 ml methanol, acidified by dissolving in HCl, and filtered by syringe filter. The filtered sample was injected in HPLC stream. Phenolics and flavonoids were identified by recording their retention time and peaks.

### 2.4. Antioxidant Activity Assay

#### 2.4.1. DPPH Free Radical Scavenging Assay

The antioxidant potential of methanol and n-Hexane extracts of M-Mln and PKM1 seeds was checked by determining the scavenging activity of DPPH free radicals based on method of Hossain et al. [41] with slight modification. 1 mL of DPPH (Sigma-Aldrich) solution was prepared. 55 *μ*L of extracts was mixed in Dimethyl Sulphoxide (DMSO), and it was further dissolved in 150 *μ*L of DPPH. The solution was then reconstituted in methanol (0.1 mM), and the final volume was made up to 250 *μ*L. The mixture was then placed in dark for 30 minutes to observe color change, and absorbance was taken at 540 nm with a spectrophotometer. The blank was run concurrently containing DMSO. The experiment was carried out in triplicate. Free radicals scavenging activity was calculated using the following formula:

(1) $$\begin{array}{c} \text{inhibition rate}\left(\%\right)=\left({\text{Abs}}_{\text{control}}-{\text{Abs}}_{\text{sample}}\right)\times \frac{100}{{\text{Abs}}_{\text{control}}}. \end{array}$$

The 50% inhibitory concentration (IC50) was calculated to evaluate the minimum active quantity of the extracts required to react with a half quantity of DPPH free radicals.

#### 2.4.2. Total Flavonoids Content

The TFC of M-Mln and PKM1 varieties of *M. oleifera* seeds methanol and n-Hexane extracts were evaluated by protocol of Sharma et al. [42] with slight modification. The extract was mixed with 2 mL of water and 0.15 mL of sodium nitrate solution, and it was incubated in an incubator for 6 minutes. Then, 4% NaOH solution was added to the mixture. The final volume was made up to 5 mL by adding methanol. Catechin was taken as a reference and standard compound. The absorbance was measured at 415 nm after the incubation in a double beam UV-Vis spectrophotometer. The total flavonoids content of the extract was expressed as catechin equivalents from standard curve of the catechin.

#### 2.4.3. Total Phenolic Content

The TPC of methanol and n-Hexane extracts of M-Mln and PKM1 varieties of *M. oleifera* seeds were assessed with Folin-Ciocalteu assay [43] with slight modification. To make a standardization curve at 0.5, 1.0, 1.5, 2.0, 2.5, 3.0, and 3.5, and 4.0 mL of gallic acid equivalent, stock solution was poured in100 mL flask. It was further mixed with distilled water to make gallic acid and sodium carbonate solution. The concentrations of phenols were checked by using reagent at 650 nm. The gallic acid was used as a standard, and thus total phenolic concentrations were expressed in the form of gallic acid equivalents.

## 3. Results and Discussion

### 3.1. FTIR Spectroscopy

The FTIR analysis, a reliable and sensitive technique, was done to detect various bonds and stretches and functional groups based on peak values in IR region [44]. FTIR spectra was obtained by using a Bruker, vector using KBr pellets at room temperature with wavenumber measured in frequency range of 4000-500 cm^−1^. The obtained peak ratio was used to separate and identify the functional groups. The FTIR spectra of M-Mln variety was recorded and the characteristic peaks (Figure 1). Most of the peaks represent major functional groups present in M-Mln variety and presents a comprehensive outlook on the presence of proteins, carbohydrates, and lipid components in the sample. A sharp peak at the 2920 cm^−1^ and 2850 cm^−1^ can be attributed and related symmetrical and asymmetrical C–H stretch [45]. Another sharp peak at 1640 cm^−1^ can be attributed to the presence of *C* = *O* bond. An amide vibration also appeared at 1420 cm^−1^.

The broad-band centered at 3420 cm^−1^ can be assigned to the presence of protein and fatty acids [45] (Figure 2). Additionally, the peak in the region of 1370 cm^−1^ is due to the combination of deformation of methyl and methylene groups [46]. Another peak at 1030 cm^−1^ can be related to the presence of carbohydrates due to *C* = *O* stretch. Furthermore, the peaks at 1300 cm^−1^ can be attributed to the low-molecular-weight carbohydrates as this region is commonly characterized as fingerprint region [47]. Moreover, the appearance of specific peaks at 3350 cm^−1^ confirmed the presence of phenolic compounds [48], signifying the antioxidant potential of seeds.

The characteristic peak values, bonds, stretches, and functional groups of both varieties are illustrated in Table 2. 13 peaks can be observed through the spectrum of M-Mln seeds sample. The corresponding peaks revealed the presence of high content of proteins and lipids in M-Mln seeds. Whereas, the spectrum of PKM1 sample showed 7 peaks of functional groups which can be related to the proteins and lipids as possible nutrients. The presence of characteristic peaks in the spectra of both varieties exhibited the presence of phenolics as well as flavonoids. These readings show that M-Mln seeds can be used as rich source of proteins and lipids due to the presence of comparatively more functional groups than that of PKM1, indicating that the indigenously produced M-Mln seeds may be an ideal source of pharmaceutical uses.

### 3.2. HPLC

HPLC is one of the most promising analytical methods used to identify and quantify different antioxidants present in plants. During this study, HPLC was used to identify the antioxidants in the methanol extracts of both varieties of *M. oleifera* seeds due to its high resolution, faster evaluation, better compound separation, and high sensitivity. The HPLC chromatograms of both varieties were successfully developed by using reverse phase column. The mobile phase at high resolution was used to obtain different peaks to quantify these compounds. Various phenolics, such as gallic acid, catechin, chlorogenic acid, coumaric acid, and sinapic acid were detected in M-Mln variety chromatogram, while quercitin was detected as flavonoid (Figure 3). Additionally, PKM1 variety chromatogram exhibited the presence of sinapic acid and salicylic acid along with coumaric acid and caffeic acid (Figure 4). The presence of phenolics and flavonoids revealed that the methanol extracts of both varieties are good source of antioxidants. The peaks of HPLC chromatogram of M-Mln variety seed methanol extract showed that it consists of high content of phenolics and flavonoids.

Caffeic acid was detected in highest amount among all the phenolics. Caffeic acid is known for its most potent antioxidant activity. The amount of phenolics can be ordered as caffeic acid > ferulic acid > gallic acid > BHT > sinapic acid > P − coumaric acid > catechin > chlorogenic acid (Table 3). Quercitin was the only flavonoid detected through HPLC chromatogram. Quercitin is one of the most potent antioxidant and also used commercially in pharmaceutical purposes. Moreover, it is a potent and versatile antioxidant, medically used to protect the cells from injury induced by inner or outer stimuli. The anti-inflammatory and antioxidant properties of phenolics and flavonoids help to remove free radicals and provide protection against free radical damage.

The maximum amount of chlorogenic acid as phenolic was detected in PKM1 seeds (Table 4). The amount of phenolic can be ordered as: chlorogenic acid > coumaric acid > caffeic acid. The amount of flavonoid in PKM1 seeds can be orderd as: sinapic acid > salicylic acid. The salicylic acid is one of the most explored and commercially used flavonoid for its antioxidative properties. Both varieties possess good amount of phenolic and flavonoid. M-Mln contains more phenolics than PKM1. HPLC analysis of methanol extract of both varieties can allow the researchers to adjust the nutritional proportions for clinical uses as antioxidants as M-Mln seeds are rich source of antioxidants specifically phenolics. Therefore, the use of moringa seeds as natural antioxidants could prove more beneficial than the synthetic and commercially available antioxidants.

### 3.3. Antioxidant Activity Assay

#### 3.3.1. DPPH Assay

DPPH radical scavenging assay is commonly used to determine the antioxidant potential, and only the potent antioxidant candidate can promisingly scavenge the DPPH free radicals, thus it may also inhibit major mechanisms associated with oxidative stress, mainly caused by lipid peroxidation. In order to evaluate the DPPH radical-scavenging activity of the two extracts of *M. oleifera* seeds, we examined a significant (*p* < 0.05) decrease in the concentration of DPPH free radicals through our specific experimental setup, due to the scavenging potential of these extracts (Figure 5).

Free radicals scavenging activity of methanol and n-Hexane extracts of M-Mln and PKM1 seeds were compared. The results were expressed as percentage of inhibition (%). The highest percentage of inhibition and least IC50 of all samples were recorded (Table 5). The highest mean percentage of inhibition of DPPH free radicals was observed in methanol extracts as compared to the n-Hexane extract of M-Mln seeds as reported by [52]. The results of DPPH free radical scavenging activity indicated that *M. oleifera* seed extracts have significant and concentration-dependent scavenging activity with the methanol fraction being the most active one as shown in Figure 5.

The results showed that the methanol M-Mln seed extract possess the highest percentage of inhibition with 60.22 ± 1.32% and followed by the methanol PKM1 seed extract which possess the percentage of inhibition of 54.92 ± 1.13% (Table 5). Though, the lowest inhibitory concentration (IC50) was 84 *μ*g/ml detected in methanol M-Mln seed extract. Many researches have revealed the effectiveness of *M. oleifera* as a source of antioxidants as evidenced by identification of Ascorbic acid, flavonoid, tocopherols, and phenolic [43, 53–55]. These findings concluded the M-Mln seeds as an excellent source of natural antioxidants.

As illustrated in Table 5, methanol extract of M-Mln seeds showed the lowest IC50 values (84 *μ*g/ml), which correspond to the greatest DPPH radical scavenging potential, followed by IC50 value of PKM1 (540 *μ*g/ml). Consistent with the reported studies, the DPPH free radicals can be effectively inhibited by methanol extract of *M. oleifera* seeds with an excellent inhibition of 60.22%, whereas the hexane extracts showed comparatively less DPPH scavenging potential, and respective percentage inhibitions were 34.53% and 29.13% at the same concentration. The radical scavenging ability of *M. oleifera* seeds is remarkable to inhibit the oxidative stress.

#### 3.3.2. Total Flavonoids Content

The antioxidant activity of extracts is mainly associated with the active phytochemicals, ubiquitous in plants. Flavonoids, a special class of phenolic compounds, can scavenge/delay the oxidation via transfer of electrons to radicals. Flavoinoids are secondary metabolites, enhance the activity of Vitamin C, biologically active and important antioxidants. In this study, TFC was done to quantify the antioxidants in *M. oleifera* seeds extracts (Figure 6). It could be seen that the methanol extract of M-Mln seeds showed the highest TFC, followed by methanol extract of PKM1. These findings were consistent with reported higher radical scavenging efficiency.

The total flavonoids content was higher in both methanol seed extracts than n-Hexane extracts (Figure 6). The methanol extract of M-Mln was found to comprise thrice flavonoids of hexane extract. Whereas, the least was observed from the n-Hexane extract of PKM1 (Table 6) as reported by [56]. The methanol extract of M-Mln was found to show highest TFC as 76.07 ± 1.10 mg/g. The hexane extract of PKM1 was found to show least TFC as 22.47 ± 1.70 mg/g.

These findings indicated that the TFC in methanol extracts were significantly higher than that of other extracts. Methanol extracts exhibited most potent radical-scavenging activity, consistent with other studies, in which the role of flavonoids as antioxidants had previously suggested. Furthermore, the antioxidant activity in plants is mainly contributed by their phenolic compounds, such as flavonoids, therefore, such findings could play a pivotal role in corresponding medicinal plants.

#### 3.3.3. Total Phenolics Content

The antioxidant efficacy of phenol-based antioxidants is mainly linked to the redox properties of the compounds and their structural characteristics such as hydrogen-donating hydroxyl groups, which ultimately afford the quenching of free radicals generated in response to oxidative damage. TPC of methanol extracts of M-Mln was found to be higher than hexane extracts (Figure 7) as the findings of [57].

The methanol extract of M-Mln was found to show highest TPC as 33.83 ± 1.19 mg/g. The hexane extract of PKM1 was found to show least TPC as 27.28 ± 0.95 mg/g (Table 7). It is due to the difference in polarity of two solvents used during study. The phenolics can be extracted in polar solvents. The results indicated the presence of fine phenolics in M-Mln variety than PKM1 variety.

Solvent based extraction of seeds has shown substantial role in varied antioxidant activity depending on their phenolic content extracted. Hydroxyl (OH) group in phenolics may be directly involved in enhanced antioxidant activity and a key determinant of their free radical scavenging ability. Nevertheless, phenolics have been reported as a significant class of secondary metabolites which are found in medicinal plants. Thus, *M. oleifera* can be used as a source of phenolics. However, its use can help to reduce the risk of diseases by its antioxidant power.

## 4. Conclusion

This study has showed that the seeds of *M. oleifera* is a potent source of antioxidants. Two indigenously produced varieties were analyzed. The antioxidant activity was greatly affected by the solvent used for extraction. The methanol extracts of both varieties showed better free radical scavenging activity than those of hexane extracts. These findings verified and validated the traditional use of seeds in order to treat oxidative stress related diseases as well as other diseases. The methanol extract of M-Mln variety with lowest IC50 value proved its more antioxidant potential than hexane extract. Besides, the total phenolics as well as flavonoids content also proved better potential of methanol extracts over hexane extracts, which contributed to antioxidant activity. Phenols and flavonoids are naturally found secondary metabolites in medicinal plant, which are extracted to cure various diseases related to oxidative stress caused by free radicals. These findings showed that the *M. oleifera* seeds possess the potency to cure oxidative stress, which can be ascribed to the presence of important phytochemicals. Thus, the present work along with previous researches reveal that the *M. oleifera* is a tremendous plant for its biomedical applications, which can be used to improve the health concerns along with overall nutrition rate in developing countries due to its nutritional benefits and biologically active products. Further work is needed to carry out more pharmacological support behind its use for its antioxidant purposes.

## Figures and Tables

**Figure 1:** FTIR spectrum of M-Mln variety seeds.

**Figure 2:** FTIR spectrum of PKM1 variety seeds.

**Figure 3:** HPLC spectrum of compounds from methanol extract of M-Mln variety *M. oleifera* seeds.

**Figure 4:** HPLC spectrum of compounds from methanol extract of PKM1 variety *M. oleifera* seeds.

**Figure 5:** Percentage of inhibition of free radicals by seed extracts of *M. oleifera*.

**Figure 6:** Total flavonoid content of extracts of *M. oleifera* seeds (mg CAE/g).

**Figure 7:** Total phenolic content of extracts of *M. oleifera* seeds (mg GAE/g).

**Table 1:** Comparative analysis of various phytochemicals and their uses isolated from different parts of *Moringa oleifera.*

Part of *Moringa oleifera*	Identified compounds	Benefits	References
Seeds	Proteins, fats, carbohydrates, amino acids (methionine, cysteine), cationic proteins, Rhamnose (4-(*α*-L-rhamnopyranosyloxy)-benzylglucosinolate), benzylglucosinolate, moringyne, monopalmitic acid, dioleic triglyceride, vitamin A, beta carotene, pterygospermin	Decrease lipid peroxides, water treatment, and antirheumatism	[11, 18–20]
Flowers	D-mannose, polysaccharide, proteins, D-glucose, and ascorbic acid	Cholagogue, aphrodisiac anti-inflammatory; cures muscle diseases, antitumor, antihysteria; stops enlargement of spleen; lower serum cholesterol level; controls lipid level of liver, and heart	[21, 22]
Roots	4-(*α*-L-rhamnopyranosyloxy)-benzylglucosinolate and benzylglucosinolate	Laxative, rubefacient, circulatory tonic; treat kidney and back pain; antifertility, antirheumatism, and antiarthritis	[14, 23, 24]
Leaves	Glycosides, kaempferol-3-O-glucoside, quercetin, 4-[4-O-acetyl-(*α* -L-rhamnosyloxy) benzyl] isothiocyanate, niazirin, niazirinin, three mustard oil glycosides, niaziminin A and B, and 3-caffeoylquinic	Full of nutrition; headache reliever; treat fever; helps in curing piles; cures throat, eyes, and ears infections; cure scurvy; control blood glucose levels	[10, 11, 18]
Gum	L-arabinose, D-mannose, D-galactose, L-rhamnose, leucoanthocyanin, D-glucuronic acid, and D-xylose	Treats dental problems; relieves headache; abortifacient; treats syphilis, and cures rheumatism; prevents dysentery; relieves intestinal pain	[25–27]
Bark	4-(*α*-L-rhamnopyranosyloxy)-benzylglucosinolate	Aids in treatment of delirium; cures eye infections; soothes earaches; work as a painkiller.	[28–30]

**Table 2:** FTIR peak values and functional groups of both varieties of seeds [48–51].

S. no	Accessions	Wavenumber (cm^−1^)	Assignment	Possible nutrient type
1	M-Mln	608	CH out-of-plane bending vibrations	Organic compounds
		935	Carbon-related component	Organic compounds
		1047	C-O stretching coupled with C-O bending of the C-OH	Carbohydrates
		1160	CO stretching, stretching vibrations of hydrogen-bonding C-OH groups	Proteins
		1235	Asymmetric PO_2_- stretching	Amide III
		1456	Asymmetric CH_3_ bending modes of the methyl group	Proteins
		1633	C-C stretch	Proteins
		1648	*C* = *O*, *C* = *N*, and N-H stretching vibrations	Proteins
		1749	Ester group (*C* = *O*) vibration of triglycerides	Lipids
		2348, 2859	NH component	Lipids
		2932, 2956	Asymmetric stretching vibration of CH_3_ of acyl chains	Lipids

2	PKM1	738	C-cl stretching vibration	Aliphatic chloro compounds
		1160	C-O bending vibration	Proteins and carbohydrates
		1270	Aryl-O stretching vibration	Aromatic ethers
		1402	Symmetric stretching vibration of COO- group of amino acids	Proteins
		1524	Stretching vibrations of *C* = *N*, *C* = *C*, and *C* = *N*	Proteins
		3093, 3275	C-H ring	Aromatic compounds

**Table 3:** Characteristic absorption peaks with their amount of M-Mln variety.

Peaks	Retention time (min)	Component	Nature	Area	Height	K-factor	Total amount (ppm)
1	2.806	Gallic acid	Phenolic	544,037.4	71,328.6	0.0007	380.82618
2	3.386	Catechin	Phenolic	338,226.6	49,771.5	0.000254	85.909
3	5.227	Chlorogenic acid	Phenolic	104,856.7	11,091.5	0.000556	58.3003
4	5.596	P-coumeric acid	Phenolic	116,404.2	12,438.0	0.000871	101.388
5	7.041	BHT	Phenolic	762,383.8	80,103.7	0.00025	190.595
6	7.842	Caffeic acid	Phenolic	1,318,761.3	70,615.5	0.00040	527.50
7	12.679	Sinapic acid	Phenolic	344,898.5	33,079.7	0.000435	150.030
8	12.967	Ferulic acid	Phenolic	542,153.2	51,932.4	0.000877	475.46
9	24.893	Querctin	Flavonoid	270,762.4	20,610.2	0.000665	180.05

**Table 4:** Characteristic absorption peaks with their amount of PKM1 variety.

Peak	RT (min)	Component	Nature	Area	Height	K- factor	Final amount (ppm)
1	2.799	Chlorogenic acid	Phenolic	484,088.1	53,554.5	0.0008	387.27
2	3.023	Coumaric acid	Phenolic	537,838.6	62,551.3	0.0001	53.7838
3	7.478	Caffeic acid	Phenolic	73,891.8	4,703.5	0.0004	29.556
4	12.176	Sinapic acid	Flavonoid	1,039,867.8	70,823.3	0.0003	311.96
5	15.608	Salicylic acid	Flavonoid	34,881.7	2,630.1	0.00023	80.2227

**Table 5:** Mean (%) inhibition of DPPH radicals of M-Mln and PKM1 seeds *of M. oleifera*.

Extract	Samples	Mean (%) inhibition of DPPH radicals ± SD	IC50 (*μ*g/ml)
Methanol	M-Mln	60.22 ± 1.32	84
	PKM1	54.92 ± 1.13	540

Hexane	M-Mln	34.53 ± 1.51	
	PKM1	29.13 ± 1.24	

*n* = 3 means values represent mean percentage inhibition of DPPH radicals of M-Mln and PKM1 seeds of *M. oleifera.*

**Table 6:** Total flavonoid content of extracts of *M. oleifera* seeds.

Extracts	Samples	TFC of *M. oleifera* (mg CAE/g)
Methanol	M-Mln	76.07 ± 1.10
	PKM1	53.75 ± 0.90

Hexane	M-Mln	42.68 ± 2.12
	PKM1	22.47 ± 1.70

*n* = 3 represents mean values of TFC of *M. oleifera* seeds.

**Table 7:** Total phenolic content of *M. oleifera* seeds.

Extracts	Samples	TPC of *M. oleifera* seeds (mg GAE/g) mean SD
Methanol	M-Mln	33.83 ± 1.19
	PKM1	32.07 ± 1.13

n-hexane	M-Mln	27.69 ± 1.50
	PKM1	27.28 ± 0.95

*n* = 3 represents mean value of *M. oleifera* seeds.

## Data Availability

There is no data availability for this manuscript.
